The article "Prediction Value of Epilepsy Secondary to Inferior Cavity Hemorrhage Based on Scalp EEG Wave Pattern in Deep Learning" was retracted in 2023. Reasons: signs of a paper mill; suspected computer-generated content; unreliable results or conclusions; concerns about the data.

# Prediction Value of Epilepsy Secondary to Inferior Cavity Hemorrhage Based on Scalp EEG Wave Pattern in Deep Learning

**DOI:** 10.1155/2022/2084276

**Published:** 2022-03-15

**Authors:** Shishuang Jiang, Xuenong He

**Affiliations:** ^1^Department of Critical-care Medicine, Yongchuan Hospital Chongqing Medical University, Yongchuan, Chongqing 402160, China; ^2^Department of Neurosurgery, Yongchuan Hospital Chongqing Medical University, Yongchuan, Chongqing 402160, China

## Abstract

**Objective:**

To search the predictive value of epilepsy secondary to acute subarachnoid hemorrhage (aSAH) based on EEG wave pattern in deep learning.

**Methods:**

A total of 156 cases of secondary epilepsy with lower cavity hemorrhage in our hospital were selected and divided into the late epilepsy group and the early epilepsy group according to seizure time, and the nonseizure group and the seizure group according to seizure condition. General data of patients were collected, the EEG types of each group were analyzed, and the disease recurrence rate, treatment effect, and symptom onset time were compared.

**Results:**

Rapid and slow and rapid blood flow velocity were the main abnormal manifestations of epilepsy secondary to inferior cavity hemorrhage, accounting for 33.3% and 18.6%, respectively. Compared with the seizure group, the proportion of type ii and type iii in the nonseizure group was higher, and the proportion of type ii and type iii in the early epilepsy group was higher than in the late epilepsy group (*P* < 0.05). The diagnostic accuracy, missed diagnosis rate, misdiagnosis rate, specificity, and sensitivity of the EEG wave pattern were 94.9%, 3.2%, 1.9%, 91.7%, and 96.2%, respectively. Compared with the early epilepsy group, the recurrence rate of type iii and type iv in the late epilepsy group was higher (*P* < 0.05). The effective rates of the attack group and the nonattack group were 72.7% and 97.0%, respectively. Compared with the attack group, the effective rate of the nonattack group was higher (*P* < 0.05). The effective rates of the early epilepsy group and the late epilepsy group were 91.7% and 85.0%, respectively. Compared with the late epilepsy group, the effective rate of the early epilepsy group was higher (*P* < 0.05). Compared with the early epilepsy group, the late epilepsy group had longer tonic-clonic seizures, atonic seizures, and absent seizures, and the difference between the groups was statistically significant (*P* < 0.05).

**Conclusion:**

In aSAH secondary epilepsy disease prediction, based on indepth study of the scalp EEG wave type prediction, they play an important role, including aSAH high-risk secondary epilepsy wave types for V, III, and IV types, as well as early and late epilepsy associated with disease stage. Through the diagnosis method to predict the severity of disease, this builds a good foundation for clinical treatment. It is beneficial to improve the effective rate of treatment.

## 1. Introduction

The aSAH refers to blood inflow into the subarachnoid space and rupture of intracranial aneurysms, which is very dangerous and the main complication is epilepsy [1]. Patients with aSAH complicated with epilepsy have a higher risk of aneurysm rupture and sudden death. Although prophylactic antiepileptic drugs have been widely used in the clinical treatment of aSAH patients, their side effects are relatively high [2]. In addition, due to individual differences in patients, there are differences in the way of drug withdrawal and the duration of drug use [3]. At present, scalp electroencephalogram is commonly used in clinical diagnosis, which is characterized by low cost, simple, noninvasive, and convenient diagnosis. However, the predictive value of different waveforms for aSAH-induced epilepsy is not clear, and whether it can guide the treatment of patients is still unclear [4]. In order to more accurately analyze the predictive value of EEG wave patterns based on deep learning for epilepsy secondary to inferior cavity hemorrhage and improve the feasibility of research results [5]. In this study, 156 patients with epilepsy secondary to inferior cavity hemorrhage admitted to our hospital were selected to explore the scalp EEG wave points of different seizure conditions and seizure times, respectively, in the hope of providing a more effective reference for clinical treatment of patients, as reported below.

The control of human brain tissue on human emotions, thinking, and behavior is diverse and complex, which will affect people's normal lives and increase the scope and difficulty of diagnosis of mental diseases [6]. Patients with mental diseases have emotional and cognitive dysfunction, and the disability rate and susceptibility of chronic diseases are high. Through the establishment of an auxiliary diagnosis and treatment analysis platform for schizophrenia, as well as medical behavior guidance and research interaction, it can play an important role in improving the service capacity of hospitals in various regions, balancing medical resources and reducing doctor-patient conflicts [7]. Giving information technology, the disease classification method of objective data, which can realize the EEG data, the brain computed tomography (CT) scan data, and the human brain MRI diagnosis, can change the status of the biological potential of the brain records. Compared with the human brain MRI data, the time series of brain change more accurately reflects in stimulating brain hemorrhage and epilepsy prediction and is of great significance [8]. As early as 1924, electroencephalography (EEG) was invented. Multiple electrodes can find and record spontaneous biological points and data maps, which can realize time-domain sampling of different locations in the brain. With the continuous progress and development of medical technology, EEG technology has developed rapidly, which can record brain activities and has been widely used in neurology, human-computer interaction, and psychology [9].

## 2. Related Studies

Deep learning scalp EEG wave pattern model has a high application value in epilepsy secondary to inferior cavity hemorrhage. Some scholars have recorded the self-unity and interindividual difference of scalp EEG wave pattern model, which can be applied in personal identity authentication and individual classification of EEG. In addition, it can be combined with EEG P300 potential data and *µ*/*β* wave to achieve two-dimensional movement on the interface. By analyzing the amplitude characteristics of EEG signals by power spectrum, selecting the characteristic components of information by Fisher ratio, and combining them with online feedback, real-time control, and off-line training, subjects' intentions can be transformed into the robot and robot navigation can be realized. In addition, through visual stimulation, EEG data potential topology can perceive the brain's response to external things, which plays an important role in perception and prestimulation activities. The basic structure of the current mainstream framework includes a fully connected layer, convolution layer, normalization layer, pooling layer, and activation function. It is mainly achieved through the following steps: using the American NicoletOne system to monitor the scalp EEG waveform model and using the estimated international standard 10–20 system for electrode placement. The average reference electrode was used to record, switch the lead mode to be switched, and set the EEG analysis parameters of 0.5–70 Hz, 30 mm/s paper speed, and 7.5 *μ*V/mm sensitivity. We train the scalp EEG waveform model with an overall strategy using image patches extracted from point locations, and first train each patch-level feature extraction network individually. After the image patch-level feature extraction network is trained to converge, for each input image, we can obtain disease label-related feature vectors from the image patch corresponding to each feature point on the image. The feature vector is then applied to train the whole-brain hierarchical graph convolutional neural network, in order to reduce the difficulty of end-to-end training of the model. After the pretraining, we use the parameters obtained from the pretraining to initialize the corresponding parameters of the model, and then train the entire model execution side to strengthen the feature exchange of each part to achieve optimal parameters. Select the loss function and set it as a 10' model learning rate. Training and testing are performed on a computer with a single graphics card installed. The results were then tested, and typical cases of epilepsy secondary to inferior cavity hemorrhage were analyzed from different characteristics, as shown in Figure 1 [10].

## 3. Data and Methods

### 3.1. General Information

A total of 156 cases of epilepsy secondary to inferior cavity hemorrhage in our hospital were selected, and they were divided into the late epilepsy group and the early epilepsy group according to seizure time, and the nonseizure group and the seizure group according to seizure condition. Among 156 patients, 58 were males and 98 were females, aged 18–75 years old, with an average age of (50.2 ± 4.4) years old, including 22 cases of secondary epilepsy, 10 cases of late epilepsy, and 12 cases of early epilepsy, respectively. There were 10 cases of focal attack and 12 cases of overall attack. The subjects agreed to the study and were approved by the hospital ethics committee.

### 3.2. Inclusion Criteria

The inclusion criteria were as follows: (1) patients meeting the consensus diagnostic criteria of the international alliance against epilepsy; (2) patients with epilepsy after aneurysm rupture and hemorrhage; (3) patients with normal cognitive function who can cooperate with the study; (4) patients with stable vital signs; and (5) patients who did not participate in other relevant studies during the study period.

### 3.3. Exclusion Criteria

The exclusion criteria were as follows: (1) patients with significant EEG interference and affected study results; (2) patients with recurrent or recurrent aneurysms; (3) patients with epilepsy induced by other factors other than arterial rupture; (4) patients complicated with other cerebrovascular diseases; and (5) patients with abnormal coagulation.

### 3.4. Methods

Scalp electroencephalogram (American NicoletOne system) was used to monitor the patients' epilepsy symptoms, and the electrode system was the international standard 10–20 system. The appropriate lead mode was chosen, and the electrode condition in time was recorded. The EEG analysis parameters were set; sensitivity: 7.5 *μ*V/mm and paper walking speed: 30 mm/s. The following are the main scalp EEG waveforms of aSAH patients: type i indicates normal EEG; type ii refers to the type of slow wave electroencephalogram (EEG), which includes three conditions: unimportant tip, simple slow wave, and atypical tip; type iii denotes explosive slow wave, including sharp wave, synchronous explosive *θ*/*δ* rhythm, and so on; and type V, electrical attack type is a phenomenon of lack of objective or subjective consciousness and behavior. The time of rhythmic episodic discharge on EEG is usually longer than 10 s. The determination of EEG type and waveform should be carried out by experienced professionals. If there is any discrepancy in the results, it is necessary to explore together and record the test results in detail.

### 3.5. Observation Indicators

#### 3.5.1. General Data

The gender and age of the seizure group, nonseizure group, early epilepsy group, and late epilepsy group were statistically analyzed.

#### 3.5.2. Predictive Value of Epilepsy Secondary to Inferior Cavity Hemorrhage

The number of abnormal patients with increased blood flow velocity, slowed blood flow velocity, asymmetric blood flow velocity, turbulence, or eddy current was counted and the incidence was calculated. The diagnostic accuracy, missed diagnosis rate, misdiagnosis rate, specificity, and sensitivity were calculated.

#### 3.5.3. EEG Type

Including 5 EEG types of type i, type ii, type iii, type iv, and type V, the corresponding cases were counted and the incidence was calculated.

#### 3.5.4. Disease Recurrence Rate

The number of patients with and without recurrence was counted.

#### 3.5.5. Therapeutic Effect

Invalid: no significant improvement or aggravation of clinical symptoms; effective: clinical symptoms and blood indicators were significantly improved; and significant effect: the patient's clinical symptoms disappeared basically, and the blood indexes could be maintained within the normal range. Effective rate = (significant + effective) number of cases/total number of cases ×100%.

#### 3.5.6. Patient Prognosis Analysis

The seizure times of tonic-clonic seizures, atonia seizures, and absence symptoms were statistically analyzed.

### 3.6. Statistical Methods

The collected data were input into Excel, and the statistical software SPSS22.0 was used for data analysis. The normal distribution test was carried out on the collected data. If the data met the normal distribution, the composition ratio and rate were used to describe the counting data, and the chi-square test was used to analyze the difference between groups. The *T* test was used to analyze the difference between groups. Logistic regression was used to analyze the influencing factors of physical fitness in the case group, and *P* < 0.05 was considered to be statistically significant. The GraphPad Prism8 was used in the study.

## 4. Result

### 4.1. Analysis of General Data of the Four Groups

Gender and age data of the seizure group, the nonseizure group, the early epilepsy group, and the late epilepsy group were comparable without statistical significance (*P* > 0.05) (Table 1).

### 4.2. Predictive Value of the EEG Wave Pattern for Epilepsy Secondary to aSAH

Rapid and slow and rapid blood flow velocity were the main abnormal manifestations of epilepsy secondary to lower cavity hemorrhage, accounting for 33.3% and 18.6%, respectively (Table 2).

### 4.3. The Diagnostic Accuracy Rate of the EEG Wave Pattern for Epilepsy Secondary to aSAH

The diagnostic accuracy rate, missed diagnosis rate, misdiagnosis rate, specificity, and sensitivity of scalp EEG wave type were 94.9%, 3.2%, 1.9%, 91.7%, and 96.2%, respectively (Table 3).

### 4.4. Comparison of EEG Types among the Four Groups

Compared with the seizure group, the proportion of type ii and type iii in the nonseizure group was higher, and the proportion of type ii and type iii in the early epilepsy group was higher than that in the late epilepsy group, and the differences between the groups were statistically significant (*P* < 0.05) (Figure 2).

### 4.5. Comparison of Disease Recurrence Rates between the Early Epilepsy Group and the Late Epilepsy Group

Compared with the early epilepsy group, the recurrence rate of patients with type iii and type iv in the late epilepsy group was higher, and the difference between groups was statistically significant (*P* < 0.05) (Figure 3).

### 4.6. Comparison of Therapeutic Effects between the Attack Group and the Nonattack Group

The effective rates of the attack group and nonattack group were 72.7% and 97.0%, respectively. Compared with the attack group, the effective rates of the nonattack group were higher, and the differences between groups were statistically significant (*P* < 0.05) (Figure 4).

### 4.7. Comparison of Therapeutic Effects between the Early Epilepsy Group and the Late Epilepsy Group

The effective rates of the early epilepsy group and the late epilepsy group were 91.7% and 85.0%, respectively. Compared with the late epilepsy group, the effective rate of the early epilepsy group was higher, and the difference between the groups was statistically significant (*P* < 0.05) (Figure 5).

### 4.8. Prognosis Analysis of the Early Epilepsy Group and the Late Epilepsy Group

Compared with the early epilepsy group, the late epilepsy group had longer tonic-clonic seizures, atonic seizures, and absent seizures, and the differences between groups were statistically significant (*P* < 0.05) (Figure 6).

## 5. Discussion

### 5.1. Causes of Disease

Epilepsy is a multiple complications of aSAH, and the main factors for inducing epilepsy are as follows: (1) oxygen-free radicals and glutamate strongly stimulate the brain, resulting in synchronous abnormal discharge [11]; (2) vasospasm and obvious ischemia; and (3) insula damage, subarachnoid hemorrhage, and brain tissue edema [12]. In the late stage of subarachnoid hemorrhage, abnormal astrocyte hyperplasia and nerve cell degeneration will occur, which will inhibit network balance and destroy the excitability of normal neurons. Excessive excitability will affect the discharge of neurons in the brain and induce epilepsy [13, 14].

### 5.2. Types and Predictive Value of EEG for Epilepsy

The study analyzed the EEG types of the nonattack group and the attack group. The results showed that the proportion of type ii, iii, iv, and V in the attack group was 4.5%, 43.2%, 40.9%, and 11.4%, respectively, and the proportion of type ii, iii, iv, and V in the nonattack group was 1.5%, 79.5%, 11.2%, 7.8%, and 11.4%, respectively. In addition, the gender and age data of the four groups in this study were comparable, so the influence of patient clinical data on the study results could be excluded. The results showed that the proportions of type ii, type iii, type iv, and type V in the early epilepsy group were 8.3%, 70.8%, 8.3%, and 12.5%, respectively, and the proportions of type iii, type iv, and type V in the late epilepsy group were 10.0%, 80.0%, and 10.0%, respectively. The results showed that the type of EEG in the late epilepsy group was mainly type iv. The main type of EEG in the early epilepsy group was type iii. Relevant clinical research reports [15] that in the case of acute pathological damage to the cerebral cortex, electrolyte, neuronal ischemia, acid-base balance disorder, and hypoxia will be accompanied, which will greatly affect the stability of neuron cells, and obvious depolarization will further affect the activity of cortical neurons [16]. When the electrical activity spreads to the adjacent tissues, it will stimulate the thalamus greatly and produce an excitatory transient postsynaptic potential, which will then activate the distal or adjacent neuron groups and significantly change the neural network [17]. These mechanisms are consistent with the results of this study [18]. Another scholar [19] explored the mouse trauma model. The results showed that craniocerebral trauma can lead to diffuse or focal brain injury accompanied by significant abnormal electrical activity. Furthermore, the transmission of abnormal electrical activity in the thalamus, related cortex, and limbic system was further analyzed at the cellular level and molecular structure level to prolong the duration of epileptiform electrical activity, but the incidence of behavioral epileptic activity was very low [20]. Nevertheless, with the progression of the disease, there will be cerebral softening foci and astrocyte transformation, which will produce repeated stimulation to cortical cells and obvious abnormal electrical activity, increasing the sensitivity of epileptic seizures, and patients will present a series of epileptic symptoms [21]. Therefore, accurate prediction methods should be explored clinically [22, 23]. In this study, the scalp EEG wave pattern prediction of patients with epilepsy secondary to inferior vena-cava hemorrhage is based on deep learning, and the patient's condition can be comprehensively predicted by increasing, decreasing, and increasing blood flow rate. The results showed that the diagnostic accuracy, missed diagnosis rate, misdiagnosis rate, specificity, and sensitivity of scalp EEG waveform were 94.9%, 3.2%, 1.9%, 91.7%, and 96.2%, respectively. Compared with head MRI and CT diagnosis, the scalp EEG waveform prediction method based on deep learning has a relatively higher prediction value and is easy to operate, which can identify the types of diseases and then analyze the prognosis of patients.

### 5.3. Analysis of Relapse of Epilepsy

Epilepsy patients also have a latent period, with obvious spike discharge and seizure characteristics. The study analyzed the recurrence rate of patients. The results showed that compared with the early epilepsy group, the recurrence rate of patients with type iii and type iv in the late epilepsy group was higher (*P* < 0.05). Therefore, the withdrawal time should be selected under the guidance of EEG, and the withdrawal time should not be stopped privately. The compliance of patients with medication can be improved through health education [24]. Some scholars [25] analyzed the problems related to seizure latency through the mouse epilepsy model. The latency from the first seizure of spontaneous epilepsy to spike wave was about 7 days, but the latency of some epilepsy patients was several months. The EEG types in this study group are mainly type iii, type iv, and type V. The results showed that seizures may be closely related to EEG stages, and it is the main type of epilepsy, which is feasible for the prognosis of the disease [26]. After treatment, the clinical symptoms of the patients were obviously relieved, and the symptoms occurred in a short time. However, there are also some patients whose treatment effects are not satisfactory. Patients should make clinical diagnoses regularly and choose the stopping time according to the diagnosis results [27].

To sum up, the scalp EEG waveform based on deep learning plays an important role in the prediction of aSAH secondary epilepsy, among which the high-risk waveform of aSAH secondary epilepsy is type V, type III, and type IV. Early and late epilepsy are related to the stage of the disease. This diagnostic method [28]can be used to predict the severity of the disease, lay a good foundation for the formulation of clinical treatment measures, and help to improve the effective rate of treatment.

## Figures and Tables

**Figure 1:** There are significant differences in the situation of inferior cavity hemorrhage in different cases, which are mainly manifested in bilateral frontal-temporal high-amplitude slow wave bursts, alpha rhythm background, and wave patterns. (a) Type ii (2–3 Hz *δ* rhythm in the right frontotemporal lead with a background of *α* rhythm); (b) type i (normal type, with a background of *α* rhythm, and without apical wave and slow wave); (c) type iv (focal slow wave in the right frontotemporal lead, typical type of apical spinous slow wave, and apical spinous slow wave); and (d) type iii (bilateral frontotemporal lead with rhythmic high amplitude slow wave eruption, background of alpha rhythm, and explosive slow wave type).

**Figure 2:** There is a significant difference in the type of disease between the epileptic seizure group and the nonseizure group. As the disease worsens, type iii accounts for a higher proportion, and the difference is statistically significant (*P* < 0.05).

**Figure 3:** The recurrence rate of the disease in the late-stage epilepsy group is higher than that in the control group, and the difference is statistically significant (*P* < 0.05).

**Figure 4:** The effective rate of treatment in the nonseizure group is higher than that of the seizure group, and the difference is statistically significant (*P* < 0.05).

**Figure 5:** The effective rate of treatment in the early epilepsy group was higher than that in the late epilepsy group, and the difference was statistically significant (*P* < 0.05).

**Figure 6:** There is a big difference in tonic-clonic seizures between the early epilepsy group and the late epilepsy group (*P* < 0.05).

**Table 1:** General data analysis of the four groups.

Group	Gender		Age (years)	*T*	*P*
	Male	Female	50.6 ± 3.6		
Attack group	11	13	51.1 ± 3.8	1.365	>0.05
Nonattack group	47	85	50.3 ± 3.3	1.054	>0.05
Early epilepsy group	5	7	50.7 ± 3.5	0.728	>0.05
Advanced epilepsy group	5	5	50.5 ± 3.2	0.637	>0.05

**Table 2:** Predictive value of EEG wave pattern for epilepsy secondary to aSAH.

Abnormal situation	The number of cases	Accounted for (%)
The blood flow rate increases	29	18.6
Slowed blood flow	27	17.3
Blood flow velocity increases and slows down	52	33.3
Flow velocity is asymmetrical	13	8.3
Turbulence	14	9.0
Total	135	86.5

**Table 3:** Predictive value of EEG wave pattern in epilepsy secondary to aSAH.

Diagnostic value	The number of cases	Accountedfor (%)
Accuracy	148	94.9
Missed diagnosis	5	3.2
The misdiagnosis rate	3	1.9
Specific degrees	143	91.7
Sensitivity	150	96.2

## Data Availability

The authors did not obtain analytical permission from the data provider because of trade confidentiality.
